This article has been retracted.

# Deep Learning-Based Networks for Detecting Anomalies in Chest X-Rays

**DOI:** 10.1155/2022/7833516

**Published:** 2022-07-23

**Authors:** Malek Badr, Shaha Al-Otaibi, Nazik Alturki, Tanvir Abir

**Affiliations:** ^1^The University of Mashreq, Research Center, Baghdad, Iraq; ^2^Department of Medical Instruments Engineering Techniques, Al-Farahidi University, Baghdad 10021, Iraq; ^3^Research Center, The University of Mashreq, Baghdad, Iraq; ^4^Department of Information Systems, College of Computer and Information Sciences, Princess Nourah bint Abdulrahman University, P. O. Box 84428, Riyadh 11671, Saudi Arabia; ^5^Department of Business Administration, Faculty of Business and Entrepreneurship, Daffodil International University, Dhaka, Bangladesh

## Abstract

X-ray images aid medical professionals in the diagnosis and detection of pathologies. They are critical, for example, in the diagnosis of pneumonia, the detection of masses, and, more recently, the detection of COVID-19-related conditions. The chest X-ray is one of the first imaging tests performed when pathology is suspected because it is one of the most accessible radiological examinations. Deep learning-based neural networks, particularly convolutional neural networks, have exploded in popularity in recent years and have become indispensable tools for image classification. Transfer learning approaches, in particular, have enabled the use of previously trained networks' knowledge, eliminating the need for large data sets and lowering the high computational costs associated with this type of network. This research focuses on using deep learning-based neural networks to detect anomalies in chest X-rays. Different convolutional network-based approaches are investigated using the ChestX-ray14 database, which contains over 100,000 X-ray images with labels relating to 14 different pathologies, and different classification objectives are evaluated. Starting with the pretrained networks VGG19, ResNet50, and Inceptionv3, networks based on transfer learning are implemented, with different schemes for the classification stage and data augmentation. Similarly, an ad hoc architecture is proposed and evaluated without transfer learning for the classification objective with more examples. The results show that transfer learning produces acceptable results in most of the tested cases, indicating that it is a viable first step for using deep networks when there are not enough labeled images, which is a common problem when working with medical images. The ad hoc network, on the other hand, demonstrated good generalization with data augmentation and an acceptable accuracy value. The findings suggest that using convolutional neural networks with and without transfer learning to design classifiers for detecting pathologies in chest X-rays is a good idea.

## 1. Introduction

Advances in data acquisition, storage, and processing allow for cheap, large-scale data collection [1]. They have improved the ability to process data into useful information and advance knowledge. This caused a substantial increase in available information in medical imaging, leaving behind the days when health data was scarce. This poses a great challenge when it comes to developing tools for its analysis and interpretation that aid in decision-making. Many modern hospitals' computer systems store a large volume of chest X-rays and radiological reports [2].

Digital image processing (DIP) allows segmentation and classification of medical images [3]. In this context, segmentation defines a partition so that the obtained regions correspond to anatomical structures, processes, or regions of special interest. Its results are used to compare volumes, morphologies, and characteristics with other studies or other regions of the same image; study tissue distribution; detect lesions; understand anatomy; plan surgeries; plan radiation therapies; and detect abnormal tissue, among other tasks. The classification requires global image analysis and helps with diagnosis and treatment.

Neural networks based on deep learning (DNN, from the English Deep Neural Network), specifically convolutional ones (CNN, from the English Convolutional Neural Networks), have seen a huge boom in recent years due to the increased capacity and availability of specific graphics processing units (GPU), the significant reduction in hardware cost, and the recent advances in machine learning [4]. In medical imaging, the number of successful DNN applications is growing [5], including organ and substructure segmentation, tumor detection, sample classification (complete images), and registration.

The automatic detection of anomalies in chest X-rays is an important application of deep learning networks in medical images that has gained momentum in the last year, due to COVID-19 detection [6, 7]. In this work, CNN automatically detects anomalies in chest X-rays from the ChestX-ray14 database [2], which contains more than 100,000 images with 14 possible pathologies. The work includes a deep study of the problem and CNN's and the development of programs for the design, training, and evaluation of networks using the Keras API on Python and GPU processing. Study, propose, implement, and validate DNN for chest X-ray anomaly detection.

## 2. Material and Methods

### 2.1. ChestX-ray14 database

The ChestX-ray14 database (Figure 1) was compiled by the NIH (National Institute of Health), the main US government agency responsible for biomedical and public health research. It comprises more than 100,000 chest X-ray images with multilabels of common diseases from more than 30,000 anonymous patients, accumulated from the year 2010 to 2020. The data was extracted from the texts of radiology reports using language processing techniques. The data set contains the following 14 varieties of abnormalities: infiltration, effusion, atelectasis, nodule, mass, pneumothorax, consolidation, pleural swelling, cardiomegaly, emphysema, edema, fibrosis, pneumonia, and hernia. Radiographs are tagged with one or more pathology keywords, resulting in single or multitags. On the other hand, the images not associated with any of the 14 classes of pathologies are labeled as “No Finding,” which is not equivalent to an image of a healthy person but could contain patterns of disease other than the 14 listed or findings uncertain within the 14 possible categories. The existence of more than one pathology associated with certain radiographs allows to analyze of the correlation between them.

### 2.2. CNNs Used in the Work

Having introduced the basic concepts of the CNNs, this subsection aims to briefly describe the architectures of the pretrained CNNs used during the development of the work; Table 1 shows some of their properties.  Figure 2 shows a general diagram of the implemented models based on transfer learning.

The proposed CNN has five convolution blocks that constitute the feature extraction phase, where 11 × 11, 5 × 5, and 3 × 3 filters are used. For its part, the qualifying phase has 2 fully connected layers, two layers of dropout, and an output layer with the same number of neurons as classes, adjusted according to the problem explored. It was decided to reduce the size of the input images to 224 × 224 pixels. Finally, the built network has 10,721,190 trainable parameters.

#### 2.2.1. VGGNet

VGGNet [8, 9] was built and trained by Karen Simonyan and Andrew Zisserman, belonging to the Vision Geometry Group (VGG) of the University of Oxford, being the winner in the location task and obtaining the second place in the classification task of the ILSVRC competition in the year 2014.

This network uses an architecture with very small convolution filters (3 × 3) achieving a significant improvement over previous CNN configurations, where large convolution filters (9 × 9 or 11 × 11 from AlexNet [10]) were used. The 3 × 3 filter is the smallest filter that can be used without losing track of left/right, top/bottom, and center between neighboring pixels.

There are variants of the VGG depending on the number of hidden layers. In this work the VGG19 is used.

#### 2.2.2. Inception (GoogLeNet)

GoogLeNet [11], also known as Inception, is a CNN developed by Google researchers. The GoogLeNet architecture presented at the ILSVRC in 2014 won first place in the image classification task, beating VGG. The depth of GoogLeNet is greater than that of VGGNet. However, the number of parameters is much less, making it a better option to optimize computational costs when available resources are limited. The input data to the network are images of dimension 224 × 224 pixels, preprocessed with an average of zero.

#### 2.2.3. ResNet

ResNet introduced the concept of residual learning to address the gradient fading problem, by adding direct connections between neurons, without adding additional parameters or additional computational complexity. In 2015, it was a winner at the ILSVRC in the image classification, detection, and localization categories and the MS COCO in the detection and segmentation categories.

ResNet introduced the residual block concept with the idea of information flowing across connections, allowing it to build much deeper networks. The residual block consists of various network layers and a direct access connection (Figure 3).

### 2.3. Regularization

When developing DNN, it is common to see overfitting, where the model works well with training data but has poor generalization. A neural network learns latent data patterns and adjusts model weights to fit them during training. This becomes complicated when the pattern he finds is just noise. Real-world training data may be affected by noise and differ greatly from real data. If a neural network is overtrained, that is, it overlearns the training data, and these contain noise, then the internal parameters probably move in their adjustment with respect to the values they would obtain in noise-free data, which means the network is less robust to noise and cannot generalize well. The pseudocolor images are segmentation results from the gray PD, T1, and T2 input images. MLP stands for multilayer perceptron. You cannot train a generalizable model when you have too few samples to learn from. If the data were infinite, the model would be exposed to all data distribution aspects, preventing overfitting Regularization decreases overfitting. Dropout and data augmentation are two DNN regularization methods.

#### 2.3.1. Dropout

The dropout technique is one of the most effective and used techniques. This method, applied to a layer, consists of arbitrarily “deactivating” (zeroing) some neurons of a layer during each training iteration. A number of output features of the layer are randomly discarded. The fraction of the features that are reduced to zero is a parameter of choice known as the dropout rate.

It can be seen in Figure 4 how the regular network (left) has all the neurons and connections between two successive layers intact, whereas, with dropout, each iteration induces some defined degree of randomness by arbitrarily deactivating or discarding some neurons and their associated connections.

#### 2.3.2. Data Augmentation

Data augmentation consists of generating more training data (in quantity and/or diversity) from the existing training samples, increasing the samples through a series of random transformations that generally consist of rotations, transformations related, translations, and scaling, among others. At the training time, the goal is that the model never sees exactly the same image twice and thus generalizes better [12], known as dynamic data augmentation (Figure 5).

### 2.4. Model Validation

Generalizability is used to evaluate a neural network's quality. To estimate generalization capacity, a suitable metric and mechanism must be defined. This work uses accuracy as the metric and hold-out as the estimation method when working with DNN.

Accuracy is the ratio of correct predictions to total predictions. It measures model generalizability. Correct generalizability estimation requires evaluating the model with untrained data. The hold-out validation method randomly creates two disjoint partitions of the original data set [13].  Figure 6 depicts hold-out.

Given that different subsampling of the data set or random initializations of the internal parameters of the DNNs can usually be used, it is common to carry out more than one entry/test cycle defining a different hold-out for each one. In these cases, the metric is obtained as the average of the values obtained over the different cycles.

### 2.5. Development Environment and Implemented Programs

Python 3.8.5, Keras 2.4.3, and TensorFlow were used to implement classification models. Python was chosen because it has many data analysis and deep learning libraries, extensive documentation, and a large programming community.

The code was structured in well-defined functions to create clear and readable code. Data loading and preprocessing functions were defined to obtain the necessary data sets for each proposed experimental arrangement, separate training and test data, generate tensor image batches with real-time data augmentation, create classification models and adjust them, graph results, and analyze them. The code was designed to be reused in each experiment with adequate documentation, saving time and reducing redundancy.

Jupyter Notebook, a 2015 client-server application, was used to develop the codes. A Jupyter Notebook is a “computational narrative” that publishes code and data with analyses, hypotheses, and conjectures. “.ipynb” files are simple, documented JSON files. It was chosen because it was accessed through a web browser, allowing the same interface to run locally as a desktop application and on a remote server [14, 15].

Jupyter Notebook was run on a remote server at the ICyTE Image Processing Laboratory using a local web browser and SSH. SSH encrypts client-server connections. Authentication, commands, output, and file transfers are all encrypted.

Conda was a package manager and environment manager. Conda lets you run different versions of Python and its libraries in virtual environments. The work was done in a virtual environment separate from other projects.

Since deep learning training takes a long time, Screen or GNU Screen was used to keep remote sessions active. It is possible to start a screen session, open multiple virtual terminals, and then log out while the processes continue. By establishing a new connection, terminals can be accessed without interrupting processes [12, 13].

#### 2.5.1. Obtaining New Data Sets from the Original Data Set ChestX-ray14

Different experimental designs required new data sets from the original database. The open-source libraries NumPy, which manages vectors and matrices in Python, and Pandas were used to obtain these sets.

In this case, the ChestX-ray14 CSV file containing class labels, image paths, radiograph information, and patient information was used. We used the radiograph paths and labels for the proposed analysis, discarding unnecessary data. Only in experiment #1 was radiograph orientation preserved. The main challenge was creating functions for each problem.

The labels had to be pure in #2 and #4; the radiographs had to show a single pathology. In this case, functions were programmed to filter the database by label. Fix #1 used this function to filter images by orientation. To fix #3, all pathological X-ray images (whether pure or not) had to be relabeled as “finding,” generating a new data set with the categories “no finding” and “finding.” A program was developed for this.

Unbalanced data was one of the work's greatest challenges, so experimental arrangement #2 was proposed. A data balancing function was programmed to obtain the number of pure pathological samples and subsample the majority class until the minority class number was equal. Reusing the same function for “pure pathology” and “no finding” In array #4, the same logic was used to obtain X-ray images labeled with a single pathology by subsampling the set without substitution.

All cases required a single data set. Multiple sets were obtained in cases where filtering was used, each group belonging to each filtered category (15 categories for array #2 and pure labels with a frequency of 500 or more for fix #4). Therefore, the sets are needed to be concatenated.

The Pandas library's concatenation function created a new data set with the labels in the same order as the individual sets. Balancing cannot be ensured in partitions performed after a concatenation using this library, which harms the generalization capacity of the models and, consequently, the quality of the experiment and conclusions drawn. Programming a function to partition and concatenate data sets preserved class balance.

#### 2.5.2. Image Batch Generation

The preprocessing API in the Keras library has classes and functions for working with images that help convert raw data on disc into an object that can be used to train a model. It was used to both preprocess the input data and apply data augmentation to it.

The ImageDataGenerator class, also known as a generator, allows you to set parameters for preprocessing input data before feeding it to a model. On the one hand, this class was used in the experiments with pretrained CNNs, and the same preprocessing that was used in ResNet, VGG, and Inception was applied to the set of radiographs. The gray levels of the radiographs were normalized to the interval [0.1] for the proposed architecture without transfer learning. Specific functions were programmed in each case.

Most deep-learning classification data sets organize all of the images into separate directories labeled with the names of the classes, making it simple to read the images from the disc. This is not the case with ChestX-ray14, where all images are stored in a single directory and their tags are mapped to a CSV file, as described in the previous subsection.

The method flow from the data frame of the ImageDataGenerator class was used to generate the image batches, which allows the data frames generated with the data set generation functions [16] to be used as input parameters. The method returns an iterator that generates tuples (*x*, *y*), where *x* is an array of batches of tensor images and *y* is a vector containing the labels. The batch size refers to the number of images used in each training step before a model's trainable parameters are updated. Because the GPU's memory is limited, a batch size of 128 images was chosen, with a validation set of 256 images. Specific functions were created as a result of this stage to define batches to be used in the training and evaluation of the models.

*(1) Augmenting Data with the ImageDataGenerator Class*. The ImageDataGenerator class also allows you to apply data augmentation. Keras augmentation is focused on generating diversity in the data shown to the model from epoch to epoch, maintaining the original amount of data. By instantiating the ImageDataGenerator class, transformations are defined, and then, during training, batches with images transformed in real time are assembled. It seeks to make the most of the training examples so that the model never sees exactly the same image twice; this helps to avoid overfitting and the model generalizes better.

To implement data augmentation, a function was defined in such a way that it would return the instance to the ImageDataGenerator class configured to perform transformations on the data. Taking into account previous articles that analyzed chest X-ray images [10, 17–21], the following transformations were defined:

- A random rotation within the range of -5/+5 degrees
- A random horizontal and vertical shift of 5%
- A random increase range of 15%
- A random distortion along an axis of 0.1 degrees creates or rectifies the angles of perception
- A padding to keep the size of the input images constant, mirroring neighboring pixels to fill in the gaps with missing pixels

The programmed function makes use of the flow_from_dataframe method to apply the transformations defined by the generator and assemble the image batches. Dynamic data augmentation was applied during model training by calling the function at each epoch.

In order to correctly evaluate the generalization capacity of the model, data augmentation was not applied to the validation data set, so another function had to be programmed with another generator without including the transformation parameters mentioned above. In this case, the implementation uses the flow_from_dataframe method prior to classifier training to generate the image batches.

#### 2.5.3. Implementation of Classification Models Using Keras

The classification models were built with the Keras functional API [21–25], allowing for nonlinear topology models and creating more complex networks than the Keras sequential model. This API was chosen because it is extremely useful for implementing transfer learning. It can handle shared layers, which means you can access and reuse a model's middle layer activations, allowing you to use its features to create new feature extraction models that return the activation values. The weights of the convolutional layers were frozen (to avoid their adjustment during training), and the feature extraction phase was extracted for later use in transfer learning-based models.

Specific programs were written to implement both the architecture proposed and the classification phase of the models obtained from pretrained CNNs, in which the model class was used to create the model and the layers class was used to instantiate the necessary layers and define their parameters (number of neurons, activation functions, filters, filter size, type of pooling, dropout, and so on), both of which are part of the Keras library. Layers in Keras are unfrozen by default, allowing them to adjust their weights during network training.

A function was programmed to return the model. The base model and the classification scheme were used as parameters; and the number of classes according to the experimental arrangement, for the creation of the proposed architectures using transfer learning and fine-tuning. A specific function, on the other hand, was created to return the proposed architecture without transfer learning.

## 3. Results and Discussion

This section has the objective of detailing the results obtained for the experiments carried out in the work, using tables and graphs, and also to carry out an analysis of them.

First, the experimentation and analysis carried out for the selection of the base model (CNN pretrained) for the transfer learning tests are explained. Second, the results of experimental arrangements #1 to #4 for transfer learning are shown. Finally, the ad hoc CNN architecture is evaluated on the experimental arrangement that showed the best results.

### 3.1. Selection of the Base Model and Classification Scheme for Transfer Learning

In the first instance of the development of this work, a study of the classification capacity of CNN chest radiographs defined from transfer learning was carried out. Starting from the ResNet50, VGG19 and InceptionV3 pre-trained CNNs, described in the previous sections and considering the two multilayer perceptron structures of the classification phase (schemes #1 and #2).  Table 2 shows a summary of the architectures studied in the first stage of the work.

It is important to note that the experimentation was carried out equally for each proposed architecture, seeking that the results obtained are comparable. For this reason, the same hyperparameters were used for training in each of the experiments, which can be seen in Table 3.

In the search to select the best base model and the best classification scheme, the classifiers were trained by adjusting their trainable parameters with the data sets obtained for experimental arrangement #2, the classification between no finding and a specific pathology which are shown in Figure 7.

The best accuracy results were shown for architecture #1, consisting of the ResNet50 pretrained CNN and the first proposed classification scheme, as shown in Figure 8.

The differences in accuracy observed with respect to the rest of the pre-trained architectures and proposed classification schemes were not very significant, but they were minor, so it was decided to continue with the following transfer-learning experiments using architecture #1, that is, combining the ResNet50 qualifying phase and the #1 qualifying phase scheme. It should be noted that all cases presented overfitting, which will be analyzed in more detail later in this section.

### 3.2. Transfer Learning Results

#### 3.2.1. Results of Experimental Setup #1: Evaluation of Robustness in the Classification according to Orientation

After evaluating and comparing the proposed models, it was determined that ResNet50 and the multilayer perceptron #1 produced the best results in identifying pure pathologies in chest X-rays.

The problem defined in experimental arrangement #1, namely the need or not to separate the radiographs according to their orientation for subsequent classification, was investigated using ResNet50 and the classification phase scheme #1. As described in the previous chapter, the database images were filtered according to anteroposterior (AP) and posteroanterior (PA) orientation. The decision was made to perform the analysis only for the classification between “no find” and “mass” due to the lengthy computation times required for CNN training. This filtering produced two subsets, with 1544 images in the AP data set and 2734 images in the PA data set as a result of the filtering. Five training/test cycles were used to define the validation scheme.  Figure 9 summarizes the findings.

As shown in Figure 9, there is no evidence of any improvement in the average accuracy achieved. The behavior varies a lot with respect to the results obtained for the cases evaluated without filtering by orientation; although there is overfitting in both experiments, the model does not seem to improve in generalization. But on the contrary, based on the results obtained, it was decided to continue with the proposed experiments without separating the sets by the orientation of the radiographs.

#### 3.2.2. Results of Experimental Setup #2: Evaluation of Robustness in the Classification according to Orientation

Tests were carried out with the different architectures from pretrained CNNs on the data sets shown in Table 2. The results obtained in this stage of the work made evident the need to work with regularization techniques to improve the generalization of the models.  Figure 10 shows the average accuracies obtained for each case of pure pathology vs. “no finding” with and without dynamic data augmentation over 5 training/test cycles.

When using dynamic data augmentation, it can be seen that the average validation accuracy improves by more than 5% in relative terms, less for the “nodule” vs. “no finding” classification, which shows a performance degradation. The experimental results show that the use of data augmentation decreases the overfitting that was very marked from the epoch 10.

#### 3.2.3. Results of Experimental Setup #3: Classification between “Find” and “No Find”

A new data set called “Find + No Find” was created, which contains all available examples and has a total number of images of 112,120. For this experiment, the “finding” class includes all radiographs that show one or more pathologies, taking into account both simple labels and multilabels. The results obtained with and without dynamic data augmentation are 63.9 percent without data augmentation and 69.5 percent with data augmentation. There was only one training/test cycle because the data set was unique (no subsampling).

When using data augmentation for the classification between “find” and “no find,” there is no improvement in invalidation accuracy for the set. However, the results obtained in both cases are close to 70% accuracy, which is excellent given the problem's high complexity. However, when comparing the results, there is a significant improvement in overfitting when using dynamic data augmentation.

#### 3.2.4. Results of Experimental Setup #4: Classification between Different Pure Pathologies

The validation accuracy results were obtained for the average of the five training cycles of average accuracy without (27.2%) and with (28.1%) data augmentation using a set of 12 pure pathologies. The results of this experimentation were not encouraging, possibly due to the complexity of the problem posed. The use of regularization techniques did not result in any improvement in the model's lack of generalization. In terms of the validation accuracy obtained from the average of the five training cycles completed, there was a 1% improvement. However, the value obtained is close to 30% in both cases, implying that only about 3 out of every 10 radiographs shown in the model will be correctly classified. As can be seen from the results, increasing the amount of dynamic data improves the model's generalizability while reducing premature overfitting. The average validation accuracy results obtained, on the other hand, show that the proposed approach is not feasible in this experimental setup.

### 3.3. CNN Results without Transfer Learning

Based on the results obtained with transfer learning for the different experimental arrangements, it was decided to use the data set of experimental arrangement #3, composed of the labels “no finding” and “finding,” which allowed having a large number of images necessary for the training of a complete CNN.

It was decided to train the model for 300 epochs, using dynamic data augmentation and the same training hyperparameters as in the transfer learning experiments. Hold-out was performed with 80% of the data for training and the remaining 20% for testing. The training and test accuracy values for each training epoch are shown in the graph of Figure 11. As can be seen in Figure 11, the model generalizes very well, beginning to converge between epochs 150 and 200. Compared to the architecture proposed with ResNet50 and the multilayer perceptron, it shows a drastic improvement with overfitting. Likewise, the accuracy value achieved remains close to 70%, as with transfer learning.

## 4. Conclusions

This work studied deep learning models for identifying chest radiography pathologies. Scarcity of databases of this type of medical image in the public domain limits the state of the art. ChestX-ray14 has the most chest X-rays and the most research, so it was chosen for this work.

The work began with a thorough study of state-of-the-art and the adopted database's characteristics, from which different experiments were designed to test the models.

ResNet50 showed the best performance for pathology detection using CNN-based transfer learning approaches, followed by VGG19 and Inceptionv3. Transfer learning approaches allow us to affirm that this can be a valid initial strategy for using CNN in cases where there are not enough labeled images, which is common in medicine. Even with chest radiograph classification, considering the complexity of chest radiograph classification, most experiments show acceptable accuracy. Dynamic data augmentation reduced overfitting in all tests without increasing computational cost or classifier stability. The ad hoc architecture proposed to evaluate a CNN without transfer learning showed acceptable accuracy and good generalization using data augmentation, indicating it is a valid strategy to follow when available. Images are enough. DNN models with and without transfer learning proved adequate for classifying chest X-ray pathologies. The total of the programs developed in this work for the design, training, and validation of CNN, along with its documentation, is an adequate basis for the future development of a library of CNN image functions that will be added to other techniques under development in the laboratory.

## Figures and Tables

**Figure 1:** Chest X-ray images, with their respective labels, belonging to the ChestX-ray14 data set.

**Figure 2:** General architecture of the model based on transfer learning used.

**Figure 3:** Comparison between a typical CNN block and a ResNet residual block.

**Figure 4:** Illustrative figure of the dropout technique.

**Figure 5:** Dynamic data augmentation.

**Figure 6:** Simple hold-out partition of the data set.

**Figure 7:** Subsets made up of pure pathology and “without finding.”

**Figure 8:** Average accuracy results for architecture #1.

**Figure 9:** Comparison of results obtained by filtering by orientation and without filtering.

**Figure 10:** Average accuracy without and with data augmentation for the data sets made up of one pathology and “no finding.”

**Figure 11:** Accuracy vs. epoch for the CNN without transfer learning, trained with the data set composed of the labels “no finding” and “finding.”

**Table 1:** Pretrained CNN properties used in work.

Architecture	Input image size (pixels)	Depth (layers)	Parameters (millions)
VGG19	224 × 224	19	144
Inception V3	299 × 299	48	23.9
ResNet50	224 × 224	50	25.6

**Table 2:** Proposed architectures from pretrained CNNs.

Proposed architecture base model	Scheme	Multilayer perceptron
#1	ResNet50	#1
#2	ResNet50	#2
#3	VGG19	#1
#4	VGG19	#2
#5	InceptionV3	#1
#6	InceptionV3	#2

**Table 3:** Training hyperparameters used for the experiments.

Hyperparameter	Value
Optimization algorithm	Stochastic gradient descent
Loss algorithm	Cross-entropy
Times	150
Training batch size	128
Validation lot size	256

## Data Availability

The data used to support the findings of this study are included within the article.

## References

[1] Stead M., Bower M., Brinkmann B., Warren C., Worrell G. A. (2016). Large-Scale Electrophysiology: Acquisition, Storage and Analysis. *In Epilepsy: The Intersection of Neurosciences, Biology, Mathematics, Engineering, and Physics*.

[2] Wang X., Peng Y., Lu L., Lu Z., Bagheri M., Summers R. M. ChestX-Ray8: hospital-scale chest X-ray database and benchmarks on weakly-supervised classification and localization of common thorax diseases.

[3] Chauhan R., Ghanshala K. K., Joshi R. C. Convolutional neural network (CNN) for image detection and recognition.

[4] Madiajagan M., Raj S. (2019). Parallel computing, graphics processing unit (GPU) and new hardware for deep learning in computational intelligence research. *In Deep learning and parallel computing environment for bioengineering systems*.

[5] Alazzam M. B., Tayyib N., Alshawwa S. Z., Ahmed M. (2022). Nursing care systematization with case-based reasoning and artificial intelligence. *Journal of Healthcare Engineering*.

[6] Musolu M., Sadeghi Darvazeh S., Raeesi Vanani I. (2021). Deep learning and its applications in medical imaging. *In Internet of Things for Healthcare Technologies*.

[7] Jemioło P., Storman D., Orzechowski P. (2022). Artificial intelligence for COVID-19 detection in medical imaging diagnostic measures and wasting a systematic umbrella review. *Journal of Clinical Medicine*.

[8] Jwaid M. F. (2022). An efficient technique for image forgery detection using local binary pattern (Hessian and center symmetric) and transformation method. *Scientific Journal Al-Imam University College*.

[9] Sorić M., Pongrac D., Inza I. Using convolutional neural network for chest X-ray image classification.

[10] Al-Obeidi A. S., Al-Azzawi S. F. (2022). A novel six-dimensional hyperchaotic system with self-excited attractors and its chaos synchronization. *International Journal of Computing Science and Mathematics*.

[11] Abdullah Hamad A., Thivagar M. L., Bader Alazzam M., Alassery F., Hajjej F., Shihab A. A. (2022). Applying dynamic systems to social media by using controlling stability. *Computational Intelligence and Neuroscience*.

[12] Al-Baldawi A. A. A. R. (2022). The possibility of implementing industrial incubators and their role in the development of small industry and medium in Iraq. *Scientific Journal Al-Imam University College*.

[13] Muhammad B. A. M. (2022). The role of universities in developing societies by accreditation on scientific research. *Scientific Journal Al-Imam University College*.

[14] Mangeri L., Gnana Prakasi O. S., Puppala N., Kanmani P. (2021). Chest diseases prediction from X-ray images using CNN models: a study. *International Journal of Advanced Computer Science and Applications*.

[15] Stirenko S., Kochura Y., Alienin O. Chest X-ray analysis of tuberculosis by deep learning with segmentation and augmentation.

[16] Hamad A. A., Thivagar M. L., Alazzam M. B. (2021). Dynamic systems enhanced by electronic circuits on 7D. *Advances in Materials Science and Engineering*.

[17] Enbeyle W., Hamad A. A., Al-Obeidi A. S. (2022). Trend analysis and prediction on water consumption in southwestern Ethiopia. *Journal of Nanomaterials*.

[18] Ahmed I., Jeon G., Chehri A. (2022). An IoT-enabled smart health care system for screening of COVID-19 with multi layers features fusion and selection. *Computing*.

[19] Alazzam M. B., Mansour H., Alassery F., Almulihi A. (2021). Machine learning implementation of a diabetic patient monitoring system using interactive E-App. *Computational Intelligence and Neuroscience, Volume*.

[20] Ji D., Zhang Z., Zhao Y., Zhao Q. (2021). Research on classification of COVID-19 chest X-ray image modal feature fusion based on deep learning. *Journal of Healthcare Engineering*.

[21] Rahmat T., Ismail A., Aliman S. (2019). Chest X-ray image classification using faster R-CNN. *Malaysian Journal of Computing*.

[22] Qi X., Brown L., Foran D., Nosher J., Hacihaliloglu I. (2021). Chest X-ray image phase features for improved diagnosis of COVID-19 using convolutional neural network. *International Journal of Computer Assisted Radiology and Surgery*.

[23] Alazzam M. B., Al-Radaideh A. T., Alhamarnah R. A., Alassery F., Hajjej F., Halasa A. (2021). A survey research on the willingness of gynecologists to employ mobile health applications. *Computational Intelligence and Neuroscience*.

[24] Moradi M., Madani A., Karargyris A., Syeda-Mahmood T. (2018). Chest X-ray generation and data augmentation for cardiovascular abnormality classification. *Medical Imaging 2018: Image Processing*.

[25] Hammoudi K., Benhabiles H., Melkemi M. (2021). Deep learning on chest X-ray images to detect and evaluate pneumonia cases at the era of COVID-19. *Journal of Medical Systems*.

